RETRACTED

# Celiac Artery Compression Syndrome: A Rare Cause of Abdominal Angina

**DOI:** 10.7759/cureus.20011

**Published:** 2021-11-29

**Authors:** Raad A Aldahhas, Rakan M Alotaibi, Shahad S Albishi, Saud S Albishi, Heba H Nezamadeen, Hassan K Halawani, Ammar Z Faloudah, Ahmed M Abdali, Samaher H Altwirgi, Tariq H Alkaabi, Ammar M Alshareef, Mawadda O Fallatta, Mashael K Bogshan, Roqia M Alshaikh, Faisal Al-Hawaj

**Affiliations:** 1 College of Medicine, Umm Al-Qura University, Mecca, SAU; 2 College of Medicine, Imam Abdulrahman Bin Faisal University, Dammam, SAU

**Keywords:** case report, laparoscopy, abdominal angina, celiac artery, mesenteric ischemia, abdominal pain

## Abstract

Abdominal angina refers to an abdominal pain that develops shortly after food intake and gradually resolves after a few hours. It is related to insufficient mesenteric blood flow to meet the intestinal demand. In the majority of cases, this syndrome is caused by atherosclerotic narrowing of the mesenteric vessels. We report the case of a 61-year-old man, with a longstanding history of hypertension, diabetes mellitus, and dyslipidemia, who presented to the emergency department with acute abdominal pain that was aggravated by food intake. The patient reported similar but milder episodes of this pain for the last three years that led him to lose significant weight because of fear of eating. Despite this classic history of abdominal angina, his condition was misdiagnosed as indigestion, and was offered symptomatic treatment only. The basic laboratory findings were within the normal limits. The patient underwent a contrast-enhanced abdominal computed tomography scan in the arterial phase which demonstrated focal proximal stenosis of the celiac trunk due to thickened median arcuate ligament. Subsequently, the median arcuate ligament was resected laparoscopically to decompress the celiac artery. The surgical operation resulted in the complete resolution of the abdominal pain. Celiac artery compression syndrome is a rare etiology of abdominal angina. Computed tomography angiography is the imaging study of choice to make the diagnosis accurately. Laparoscopic resection of the median arcuate ligament is a safe and successful approach in the management.

## Introduction

Acute abdominal pain is one of the most frequent reasons for emergency department visits. It has a wide range of underlying pathologies. Accurate diagnosis of acute abdominal pain can be challenging [1]. Abdominal angina refers to the abdominal pain that develops after the food intake due to decreased visceral blood flow that is insufficient to meet the intestinal demands [2]. The diagnosis of abdominal angina is often delayed as the clinical manifestations are vague and non-specific. However, the classic description of abdominal angina is an abdominal pain that is out of proportion to the findings on the physical exam. The pain often develops a few minutes after eating and is gradually relieved after the next hours [3]. A high index of suspicion for this condition is crucial as none of the laboratory investigations is diagnostic. Abdominal angina can lead to significant weight loss as the patient has fear of eating because of the severe pain. The diagnosis of abdominal angina needs careful exclusion of the differential diagnoses that include peptic ulcer disease, chronic pancreatitis, chronic cholecystitis, and abdominal malignancies [4]. The majority of abdominal angina cases are related to atherosclerosis. The most important risk factor for abdominal angina includes smoking and dyslipidemia [2]. Here, we report the case of an elderly man with acute-on-chronic abdominal pain that was eventually diagnosed as a celiac artery compression syndrome, a very rare and underrecognized disorder.

RETRACTED

## Case presentation

We present the case of a 61-year-old man who presented to the emergency department with a two-day history of severe abdominal pain. The pain was generalized and non-radiating. He described the pain as burning in character and was constant. The pain was aggravated by food intake and was not relieved by over-the-counter medications. He rated the pain as 8 out of 10 in severity and he could not sleep because of the pain. The pain was associated with nausea and recurrent episodes of vomiting. The patient reported that he had been having abdominal pain that was similar in quality but much milder in severity than the current episode. He reported that he usually developed abdominal pain following meal intake. He visited several outpatient clinics for his pain. He was diagnosed as having indigestion. He has been on a proton pump therapy for two years and it has provided moderate relief to his pain. He underwent upper gastrointestinal endoscopy and revealed normal findings. He reported that because of the chronic abdominal pain, he had reduced appetite and lost more than 15 kg.

In addition to the chronic abdominal pain, the past medical history was remarkable for a longstanding history of hypertension, dyslipidemia, diabetes mellitus, and chronic obstructive pulmonary disease. The patient had a history of Helicobacter pylori gastritis 15 years back that was successfully eradicated by triple therapy. The patient was on several medications for his comorbidities, including metformin 1000 mg, amlodipine 5 mg, omeprazole 40 mg, atorvastatin 20 mg, and aspirin 75 mg. His surgical history included a remote history of tonsillectomy. He was not known to have any drug or food allergies. He was a heavy smoker with a 30 pack-years smoking history. He never consumed alcohol. He was a retired school teacher. The family history was remarkable for inflammatory bowel disease.

RETRACTED

Upon examination, the patient appeared in pain. His vital signs showed tachycardia (115 bpm), normal respiratory rate (14 bpm), normal temperature (36.8℃), and maintained blood pressure (124/91 mmHg). His oxygen saturation was normal on the room air. Abdominal examination revealed a soft abdomen with generalized tenderness. However, there was no guarding or rigidity. The bowel sounds were present and had normal intensity and frequency. Cardiovascular examination revealed a loud S2 sound with no added sounds or murmurs. The peripheral pulses were normal. The respiratory and neurological examination findings were normal. The initial laboratory findings, including hematological and biochemical investigations, were within the normal range (Table 1).

**Table 1:** Summary of the results of laboratory findings

Laboratory Investigation	Unit	Result	Reference Range
Hemoglobin	g/dL	13.1	13.0–18.0
Leukocytes	1000/mL	8.5	4.0–11.0
Platelet	1000/mL	390	140–450
Erythrocyte Sedimentation Rate	mm/hr.	14	0–20
C-Reactive Protein	mg/dL	7.5	0.3–10.0
Total Bilirubin	mg/dL	1.0	0.2–1.2
Albumin	g/dL	3.4	3.4–5.0
Alkaline Phosphatase	U/L	50	46–116
Gamma-glutamyltransferase	U/L	21	15–85
Alanine Transferase	U/L	33	14–63
Aspartate Transferase	U/L	25	15–37
Blood Urea Nitrogen	mg/dL	11	7–18
Creatinine	mg/dL	1.0	0.7–1.3
Sodium	mEq/L	137	136–145
Potassium	mEq/L	3.9	3.5–5.1
Chloride	mEq/L	104	98–107

Considering the cardiovascular risk factors for atherosclerosis and the severity of the pain, the initial differential diagnosis was acute mesenteric ischemia. Hence, the patient underwent a contrast-enhanced computed tomography scan of the abdomen. The scan demonstrated an acute angulation and indentation upon the celiac trunk with thickening of the median arcuate ligament (Figure 1). The bowel loops had normal wall thickness and enhancement. In light of the clinical and radiological findings, the diagnosis of celiac artery compression syndrome was made.

**Figure 1:** Selected axial (A) and sagittal (B) images of abdominal CT scan demonstrating focal proximal stenosis (arrow) of the celiac trunk due to thickened median arcuate ligament. CT: Computed tomography

Subsequently, the patient was prepared for surgical intervention for decompression. He underwent laparoscopic surgery. The operation was done under general anesthesia and the patient was placed in a supine position. After establishing pneumoperitoneum, diagnostic exploration was made. The thickened median arcuate ligament was appreciated. Careful dissection of the ligament was performed and the celiac artery was decompressed successfully. No complications occurred during the operation. The patient had an uneventful recovery. Postoperatively, the patient was able to tolerate oral feeding with no postprandial pain. He was discharged on the fifth postoperative day. After one year of regular follow-up visits, the patient had major satisfaction and his symptoms showed complete resolution.

RETRACTED

## Discussion

We report the case of an elderly man with acute abdominal pain due to abdominal angina that was misdiagnosed for three years. The abdominal angina was due to celiac artery compression syndrome. This syndrome develops due to compression of the proximal celiac trunk by a thickened median arcuate ligament that connects the diaphragmatic crura to the aortic hiatus. In 1965, Dunbar et al. [5] linked this anomaly to the clinical syndrome of abdominal angina. Hence, celiac artery compression syndrome is often termed Dunbar syndrome.

The diagnosis of celiac artery compression syndrome can be made after the combination of the clinical and radiological features. In contrast to abdominal angina due to atherosclerosis, celiac artery compression syndrome usually develops in young patients [6]. However, in the present case, the patient was above the age of 60 years with multiple comorbidities, suggesting that the syndrome may manifest at any age. An abdominal bruit can be heard on abdominal auscultation in the epigastric region with respiratory variation [7]. We could not appreciate this finding in our patient.

Before the era of the widespread use of computed tomography scans, the radiological diagnosis of celiac artery compression syndrome is made by conventional angiography [8]. The angiography demonstrates a superior indentation of the proximal celiac artery that is more appreciated in the expiratory phase [8]. However, it is very important to remember that some patients may have these radiological features without any clinical manifestations. Hence, the diagnosis of celiac artery compression syndrome cannot be made based on the imaging findings solely [6]. Currently, the radiological diagnosis of celiac artery compression can be established accurately by computed tomography angiography.

Regarding the management of celiac artery compression syndrome, surgical decompression is the appropriate treatment that can be made either by laparotomy or by laparoscopic approach [9]. As in the present case, surgical resection of the median arcuate ligament is often curative. However, in some patients, the thickened median arcuate ligament may induce damage to the celiac artery vasculature that requires reconstruction [6].

RETRACTED

## Conclusions

Celiac artery compression syndrome is a very rare etiology of acute and chronic abdominal pain. The diagnosis should be kept in mind in any patient with postprandial abdominal pain. Computed tomography angiography is the imaging study of choice to make the diagnosis accurately. However, the imaging findings should not be interpreted in isolation from the clinical manifestations. Surgical decompression of the celiac artery by resection of the median arcuate ligament is the treatment of choice for this syndrome. The present case demonstrated the feasibility and safety of the laparoscopic approach for this syndrome.

## References

[1] Graff LG, Robinson D (2001). Abdominal pain and emergency department evaluation. Emerg Med Clin North Am.

[2] Biolato M, Miele L, Gasbarrini G, Grieco A (2009). Abdominal angina. Am J Med Sci.

[3] Kuczyńska M, Światłowski Ł, Sojka M, Pyra K, Drelich-Zbroja A, Jargiełło T (2020). Abdominal angina: an underrecognized cause of alarming symptoms. Pol Arch Intern Med.

[4] Oliveira DM, Nunes I, Dias P (2019). Rare cause of abdominal angina. BMJ Case Rep.

[5] Dunbar JD, Molnar W, Beman FF, Marable SA (1965). Compression of the celiac trunk and abdominal angina. Am J Roentgenol Radium Ther Nucl Med.

[6] Horton KM, Talamini MA, Fishman EK (2005). Median arcuate ligament syndrome: evaluation with CT angiography. Radiographics.

[7] Muqeetadnan M, Amer S, Rahman A, Nusrat S, Hassan S (2013). Celiac artery compression syndrome. Case Rep Gastrointest Med.

[8] Fong JK, Poh AC, Tan AG, Taneja R (2014). Imaging findings and clinical features of abdominal vascular compression syndromes. AJR Am J Roentgenol.

[9] Scholbach T (2006). Celiac artery compression syndrome in children, adolescents, and young adults: clinical and color duplex sonographic features in a series of 59 cases. J Ultrasound Med.

